# Boredom Proneness on Chinese College Students' Phubbing during the COVID-19 Outbreak: The Mediating Effects of Self-Control and Bedtime Procrastination

**DOI:** 10.1155/2023/4134283

**Published:** 2023-02-08

**Authors:** Fan Meng, Bin Xuan

**Affiliations:** ^1^School of Educational Science, Anhui Normal University, Wuhu, Anhui, China; ^2^Institute of Artificial Intelligence, Hefei Comprehensive National Science Center, Hefei, China

## Abstract

**Objective:**

To analyze the relationship between boredom proneness and phubbing among Chinese college students and examine how self-control and bedtime procrastination mediate this relationship during the COVID-19 outbreak.

**Methods:**

A total of 707 Chinese college students were voluntarily surveyed. They completed the Generic Scale of Phubbing (GSP), Short Boredom Proneness Scale (SBPS), Bedtime Procrastination Scale (BPS), and Self-Control Scale (SCS).

**Results:**

(1) The results revealed that men scored higher on boredom than women. (2) The analysis revealed significant associations between each of the variables. Boredom proneness was positively correlated with bedtime procrastination (*r* = 0.318; *P* < 0.001) and phubbing (*r* = 0.418; *P* < 0.001) and negatively correlated with self-control (*r* = −0.518; *P* < 0.001). (3) Mediation analysis suggested that self-control and bedtime procrastination mediate the relationship between boredom proneness and phubbing (effect of self-control = 0.094, *P* < 0.001, 95% CI [0.062∼0.128]; effect of bedtime procrastination = 0.025, *P* < 0.001, 95% CI [0.011∼0.042]; and effect of self-control and bedtime procrastination = 0.032, *P* < 0.001, 95% CI [0.020∼0.046]).

**Conclusion:**

Self-control and bedtime procrastination mediate the association between boredom proneness and phubbing among Chinese college students during the COVID-19 pandemic.

## 1. Introduction

The COVID-19 outbreak greatly influences society by affecting both global economies and our lives as individuals. In addition to its impact on physical health, its effects on psychological health must be considered. To most, boredom is a ubiquitous experience and a unique situation for college students living and learning at home during the COVID-19 outbreak [1]. In such a setting, it is difficult for college students to avoid electronic use for many reasons, such as a lack of face-to-face communication with peers, taking classes, and browsing the Internet. Individuals with a high level of boredom may be at risk for higher levels of phubbing during the COVID-19 outbreak because they need to change their behavior to reduce boredom. Based on the literature searches conducted nationally and internationally, there is less empirical evidence on the relationship between boredom and phubbing, which is the primary significance and reason for conducting this research.

Phubbing refers to the behavior of individuals engaging with their phones during face-to-face conversations instead of talking to or paying attention to others [2]. As phubbing is a new area that has become a normalized part of everyday interactions, communication quality and satisfaction in relationships have decreased [3]. Limited but growing research into phubbing has focused on two aspects. First, phubbing negatively impacts people on relationship satisfaction and personal well-being [4]. Second, predictors of phubbing are discussed, including smartphone addiction [5], lack of self-control [6], fear of missing out [7], social anxiety [8], trait anxiety [9], and boredom [10]. Despite this, the causes of phubbing remain largely unknown. This study examined existing findings to understand factors such as boredom, self-control, and bedtime procrastination that predict phubbing. Then, a model was developed and tested to explain these factors.

Trait boredom can predict one's phubbing frequency [11], and a positive correlation has been found between boredom and phubbing [12]. Trait boredom has traditionally been described as a negative experience—a negative emotion frequently linked with difficulty sustaining attention and related impulse control difficulties [13, 14]. According to the meaning-and-attention-component (MAC) model, boredom occurs when one cannot successfully engage in an activity and/or when the current activity is perceived as meaningless [15]. As a result of the previous studies, boredom is positively correlated with several problematic behaviors, such as bedtime procrastination [16] and problematic smartphone use (PSU) [17, 18]. Therefore, it is of practical significance to explore the relationship between boredom and phubbing and which factors affect the relationship.

**Hypothesis 1 .**

Boredom proneness has a positive correlation with phubbing.

A recent study analyzing how boredom and self-control interact to guide behavior toward goals emphasizes the psychological challenges under pandemic prevention and control measures [19]. When stimulation is low during the mandatory quarantine, boredom can challenge confined college students. High levels of boredom are associated with breaking habitual behavior, such as deliberately delaying going to bed and more phubbing behaviors. Self-control plays a vital role in the relationship between boredom and phubbing. Self-control facilitates goal achievement by volitionally directing attention toward goal-directed behavior, aiming to override prepotent impulses or urges of thoughts, actions, and emotions to serve long-term goals by resisting inner desires and external temptations to adapt appropriately to the environment, which is of great societal relevance [20]. Self-control is positively associated with individuals' health, adaptive behavior, and well-being, whereas it is negatively associated with bedtime procrastination [21] and phubbing [22]. Individuals who lack self-control are more prone to addictive behaviors such as alcohol abuse [23], Internet addiction [24], and PSU [25].

**Hypothesis 2 .**

Self-control mediates the relationship between boredom proneness and phubbing.

Boredom proneness predicts bedtime procrastination [26]. Bored individuals seek activities that stimulate them more than sleeping. Trait boredom includes the concept of fidgeting, whereas fidgeting, a coping mechanism for boredom, leads to a delay in bedtime. According to the attentional theory of boredom [27], when procrastinators ignore the present moment, they are distracted from sleep and tempted to find something interesting to do, resulting in delayed bedtime [28]. Bedtime procrastination is positively related to PSU [29]. A cross-lagged analysis revealed significant bidirectional relationships between PSU and bedtime procrastination [30]. Bedtime procrastination is “failing to go to bed at the intended time with no external circumstances preventing one from doing so” and is a type of unhealthy behavior related to sleep habits [31]. The annual sleep report of China (2022) shows that only 6.41% of college students never experience bedtime procrastination [32]. However, 61.53% of them habitually play games on smartphones before going to sleep. Previous studies have shown that, instead of sleeping, up to 66.67% of college students shop on their phones, play games, chat with friends, or read novels [33].

**Hypothesis 3 .**

Boredom proneness and phubbing are mediated by bedtime procrastination.

Bedtime procrastination has been recognized as a self-control failure and a significant factor in sleep deficiency during the COVID-19 outbreak [34] and is strongly negatively related to self-control [35]. Individuals with a high level of boredom proneness will find goal achievement more challenging, and low self-control may impair their ability to handle these challenges [36]. They always give in to temptation and then delay sleep during the COVID-19 outbreak [37]. Self-control plays an essential role in PSU [38] and bedtime procrastination [39], which facilitates interpreting the relationship between boredom, bedtime procrastination, and phubbing. This study aimed to analyze the mediating effects of self-control and bedtime procrastination on this relationship.

**Hypothesis 4 .**

Self-control and bedtime procrastination sequentially mediate the relationship between boredom proneness and phubbing.

## 2. Methods

### 2.1. Participants

A random sample of adult college students was collected from three colleges in Henan Province. All participants have no history of psychiatric or neurological disease. Questionnaires, including the informed consent, were distributed through the online class community, and 713 questionnaires were returned. We removed the participants' data from the dataset if they completed the questionnaires too quickly (<5 min). Ultimately, there were 707 valid subjects with an effective rate of 99.16%, of which 211 were males (29.84%) and 496 were females (70.16%), all participating anonymously and voluntarily. The participants were between 18 and 24 years. The study was conducted in accordance with the Declaration of Helsinki. The results were analyzed anonymously.

### 2.2. Measures

#### 2.2.1. Short Boredom Proneness Scale (SBPS)

The scale was translated into Chinese and tested to measure the trait propensity for experiencing boredom for college students with excellent validity and reliability [40]. It was revised based on the original by Struk et al. [41]. It consists of eight items rated on a seven-point Likert scale. Total scores range from 8 to 56. High scores reflect general proneness to boredom. The Chinese version of the scale's Cronbach's alpha coefficient was 0.870. In this study, the value of Cronbach's alpha was 0.844.

#### 2.2.2. The Generic Scale of Phubbing (GSP)

The Chinese version of GSP among college students was revised from the original by Chotpitayasunondh and Douglas to measure the extent to which people focus on their smartphones and ignore others in social settings [42]. It is a four-factor, 15-item assessment with a seven-point Likert scale. The Chinese version of the scale's Cronbach's alpha coefficient was 0.840 [43]. In this study, the value of Cronbach's alpha was 0.870.

#### 2.2.3. Bedtime Procrastination Scale (BPS)

The Chinese version of the BPS was revised from the original by Kroese et al. [44] to measure the sleep-related behaviors and habits that could indicate levels of bedtime procrastination among Chinese undergraduates. It consists of nine items rated on a five-point Likert scale. Four items (2, 3, 7, and 9) are reverse scored. The Chinese version of the scale's Cronbach's alpha coefficient was 0.910 [45]. In this study, the value of Cronbach's alpha for the scale was 0.868.

#### 2.2.4. Self-Control Scale (SCS)

The Chinese version of the SCS was revised based on the original by Tangney et al. [46] to measure self-control among Chinese college students [47], including impulse control, healthy habits, resisting temptation, work focus, and temperance entertainment. It consists of 19 items rated on a five-point Likert scale. Except for items 1, 5, 11, and 14, all items are reverse scored, and the scores are summed to yield a total. The Chinese version of the scale's Cronbach's alpha coefficient was 0.862. In this study, the value of Cronbach's alpha was 0.849.

### 2.3. Procedure

The original data were collected through an online survey among Chinese college students. Participants were asked to complete the online survey by using Sojump (http://www.sojump.com), one of China's most professional online survey websites, within 20 minutes. This study was approved by the Anhui Normal University Institutional Review Board. The survey began on March 12, 2020, and ended on March 24, 2020.

SPSS software (version 26.0) was used for statistical analysis. First, potential common method bias was checked, and Harman's single factor test was calculated to determine the data for common method variance [48]. Second, descriptive statistics such as the means (*X*) and standard deviations (SD) for each variable were reported, followed by the correlations among focal study variables. Third, mediation analyses assessed whether self-control and bedtime procrastination mediated the relationship between boredom proneness and phubbing. A mediation analysis can use bootstrap analysis to evaluate the significance of indirect effects by using macro Process 3.3 from SPSS (version 26.0) developed by Hayes (Model 6) [49]. The lowest possible significance level was used, and the bootstrapping procedure with 10,000 bias-corrected bootstraps with 95% confidence intervals (CIs) was estimated. Bootstrapping creates an empirical representation of the population by resampling from the empirical sample to mimic the original sampling process [50].

## 3. Results

### 3.1. Descriptive Statistics and Correlation Analysis of the Variables

All items were constrained in the analysis, and the first principal factor explained only 22.14% of the variance, suggesting that common method bias is not a problem in this study. According to the results, male students had significantly higher boredom proneness than female students (*t* = 2.541; *P* < 0.05) in this study.

Partial correlations were found between boredom proneness, bedtime procrastination, self-control, and phubbing (Table 1). Boredom proneness was positively correlated with bedtime procrastination (*r* = 0.318^*∗∗∗*^) and phubbing (*r* = 0.418^*∗∗∗*^) but negatively correlated with self-control (*r* = −0.518^*∗∗∗*^). Bedtime procrastination was negatively correlated with self-control (*r* = −0.414^*∗∗∗*^) and positively correlated with phubbing (*r* = 0.402^*∗∗∗*^). Self-control was negatively correlated with phubbing (*r* = −0.448^*∗∗∗*^).

### 3.2. Mediating Effect Analysis

The mediation analysis of gender and age demonstrated that neither variable significantly impacted the relationship between boredom proneness and phubbing. The bootstrapping tests revealed that self-control and bedtime procrastination mediate the relationship between boredom proneness and phubbing (Table 2). The results indicated an effect of boredom proneness on mediating variables, −0.225 for self-control (*P* < 0.001) and 0.088 for bedtime procrastination (*P* < 0.001). Additionally, concerning the influence of mediators' variables on the outcome, the effect of self-control was −0.416 for phubbing and the effect of bedtime procrastination was 0.290 for phubbing (*P* < 0.001 in both cases).

A mediation analysis was conducted to determine the extent to which the change in phubbing was brought about by self-control and bedtime procrastination. Direct effects showed that boredom proneness had a direct positive effect on phubbing of 0.167 (*P* < 0.001), whereby the 95% bias-corrected CI did not include zero [0.111–0.224]. In addition to the direct path, there are three indirect paths: (1) the first path coefficient = *a*_1_(−0.225) ✕ *b*_1_(−0.416) = 0.094, 95% CI [0.062–0.128]; (2) the second path coefficient = *a*_2_(0.088) ✕ *b*_2_(0.290) = 0.025, 95% CI [0.011–0.042]; and (3) the third path coefficient = *a*_1_(−0.225) ✕ *d*(−0.484) ✕ *b*_2_(0.290) = 0.032, 95% CI [0.020–0.046]. The total indirect effects of boredom proneness on phubbing were significant at 0.151 (*P* < 0.001). Zero was not included in the bootstrap interval, 95% CI [0.115–0.190], suggesting that self-control and bedtime procrastination partially mediate the relationship between boredom proneness and phubbing (Table 3).

## 4. Discussion

This study explored the effect of boredom proneness on college students' phubbing and the mediating role of self-control and bedtime procrastination. The findings showed statistically significant gender differences in boredom proneness, consistent with the previous research [51]. A lack of external stimulation greatly affected men [52]. They appeared to experience greater boredom than women because men were more likely to attribute boredom to the home environment, being relatively isolated from the external world during the COVID-19 outbreak. However, women were more likely to attribute boredom to a lack of internal stimulation [53]. Furthermore, male college students experience greater boredom when they perceive their environment as lacking in activities to pursue, slow time passage, and feelings of impatience [54]. Accordingly, further research would include a more specific exploration of how segmentation dimensions of boredom influence phubbing.

According to the dual systems model of self-control [55], when faced with temptation, the reflective system prompts rational behavior for long-term goals, whereas the impulsive system prompts individuals to do what pleasure dictates [56]. Boredom proneness may be more likely to evoke activity in the impulsive system to choose hedonic behaviors, such as bedtime procrastination and phubbing. Accordingly, boredom among Chinese college students positively predicts their phubbing behaviors [57]. In contrast, the reflective system inhibits or overrides prepotent responses. In line with previous research, correlation analysis shows that self-control is negatively related to bedtime procrastination [58], phubbing [59], and boredom [60]. In contrast, phubbing is positively associated with boredom and bedtime procrastination. Results are consistent with previous studies that the higher the individual's trait of boredom is, the higher the level of phubbing is [61]. Boredom is positively related to bedtime procrastination, consistent with earlier findings that the high bedtime procrastination group spends 451% more time (about 61 minutes) per day on their smartphones before bedtime than the low bedtime procrastination group [62, 63].

The second proposition was to test the prediction that self-control and bedtime procrastination would mediate the relationship between boredom proneness and phubbing. The results of the current study can be explained according to the theorizing on the potential interplay between boredom and self-control in guiding goal-directed behavior [64]; boredom proneness and self-control play essential roles in goal-directed behavior (Figure 1). On the one hand, boredom proneness, as a signal to engage in a different activity (change behavior), should make adherence to containment measures more complicated, thus affecting bedtime procrastination and positively impacting phubbing. It indirectly affects bedtime procrastination through the mediating effect of self-control. High levels of boredom proneness can increase phubbing levels, and self-control can reduce phubbing and bedtime procrastination. Self-control is an essential intermediary variable between boredom proneness and phubbing. When boredom proneness limits reflective self-control, it increases PSU [65]. Mu's reported that self-control negatively predicts bedtime procrastination [66]. Mediating effect analysis also shows that boredom proneness can indirectly affect phubbing through the chain mediation of self-control and bedtime procrastination. A high level of boredom proneness tends to cause negative and impulsive emotions, which increase bedtime procrastination behavior among college students. Thus, they may show more phubbing behavior. However, improving self-control and reducing bedtime procrastination can reduce phubbing in college students. Concretizing existing models for the current study allows us to shed new light on how self-control and bedtime procrastination mediate the relationship between boredom proneness and phubbing.

The study has certain limitations that need to be considered. First, causal directions cannot be interpreted because the data are cross-sectional. A longer temporal dimension would reveal the evolution of self-control and bedtime procrastination and their relationship with boredom proneness and phubbing. Second, only unmarried college students participated in this research, limiting the findings' generalizability. Third, this research relied on self-reported data, often biased by social desirability and common method bias. Fourth, the current study cannot provide clear support for the reverse causal relationship between bedtime procrastination and phubbing. Finally, this model does not expound on the concrete cognitive mechanisms of phubbing.

In the future, longitudinal models need to assess the evolution of conditions in college students to understand the causal directions between phubbing and its influencing factors. The sample needs to be extended to other population groups, such as clinical or enterprise employees. In addition, to increase the diversity of participants, we encourage future research to use multi-informant approaches (such as parent reports, teacher reports, and friend reports) and mixed-method approaches. Furthermore, as phubbing and bedtime procrastination are increasing research attention, researchers need to dive deeper into the causal relationship. Future research could be extended by studies that further explain the cognitive mechanisms, particularly the cognitive mechanisms of self-control on phubbing.

These results contribute theoretically and empirically to the literature on phubbing and highlight many worthwhile questions with the hope of inspiring future research. First, based on the findings of this study, we suggested some strategies that reduce boredom, bedtime procrastination, and phubbing by training college students' self-control, time management, and commitment. Second, intervening strategies, such as the online application of mental contrast with implementation intentions [67], can reduce bedtime procrastination and phubbing, providing critical practical implications for reducing college failure. Third, metacognitive strategies enable college students to use an app to record how often they phub, rethink why they phub, and go to bed later than they intended. As mentioned above, these results provide ideas and methods for college students to carry out home-based learning. From the perspective of home-school cooperation, online training in mindfulness and home-based mindfulness practice can decrease college students' boredom [68], bedtime procrastination [69], and phubbing [70]. Furthermore, mindfulness can promote college students' self-control [71] during the COVID-19 pandemic. Mindfulness can also work against negative emotions and problematic behaviors, help students work and rest regularly, and improve the efficiency of home-based learning for college students. From the perspective of college students, the promotion function of classmate friendship can reduce boredom, and students can benefit from forming an online study group to study and live regularly. In the group, students will share their home-based learning progress and achievements to monitor and encourage each other's progress.

In conclusion, boredom proneness, self-control, and bedtime procrastination are essential factors that affect college students' phubbing, while self-control and bedtime procrastination are mediating variables affecting phubbing.

## Figures and Tables

**Figure 1:** The influence of boredom proneness on phubbing in the current study.

**Table 1:** Correlations between boredom proneness, bedtime procrastination, self-control, and phubbing.

	*M* ± SD	Boredom proneness	Self-control	Bedtime procrastination	Phubbing
Boredom proneness	3.455 ± 0.953	1			
Self-control	3.179 ± 0.414	−0.518^*∗∗∗*^	1		
Bedtime procrastination	2.969 ± 0.587	0.318^*∗∗∗*^	−0.414^*∗∗∗*^	1	
Phubbing	2.744 ± 0.728	0.418^*∗∗∗*^	−0.448^*∗∗∗*^	0.402^*∗∗∗*^	1

Notes: ^*∗∗∗*^*P* <  0.001; *M* = mean; SD = standard deviation.

**Table 2:** Results of regression analysis in the chain mediation model.

Variables		Model fitting indicator			Effect value		95% CI	
Outcome variable	Predictor variable	*R*	*R* ^2^	*F*	*B*	*t*	LLCI	ULCI
Self-control	Boredom proneness	0.518	0.269	86.132	−0.225(*a*_1_)	−15.994^*∗∗∗*^	−0.253	−0.198

Bedtime procrastination	Boredom proneness	0.432	0.187	40.249	0.088(*a*_2_)	3.562^*∗∗∗*^	0.039	0.136
	Self-control				−0.484(*d*)	−8.583^*∗∗∗*^	−0.595	−0.373

Phubbing	Boredom proneness	0.541	0.292	57.939	0.167(*c*)	5.826^*∗∗∗*^	0.111	0.224
	Self-control				−0.416(*b*_1_)	−6.056^*∗∗∗*^	−0.551	−0.281
	Bedtime procrastination				0.290(*b*_2_)	6.642^*∗∗∗*^	0.204	0.376

*Note.* ^*∗∗∗*^ *P* < 0.001; *C* = constant; CI = confidence interval; LLCI = low limit confidence interval; ULCI = upper limit confidence interval.

**Table 3:** Results of the mediation test using bootstrap analysis.

Type	Mediation paths	Estimate	Std. err	Bootstrap 95% CI	
				Lower	Upper
Indirect 1	Boredom proneness—self-control—phubbing	0.094	0.172	0.062	0.128
Indirect 2	Boredom proneness—bedtime procrastination—phubbing	0.025	0.008	0.011	0.042
Indirect 3	Boredom proneness—self-control—bedtime procrastination—phubbing	0.032	0.007	0.020	0.046
Total indirect		0.151	0.019	0.115	0.190
Direct	Boredom proneness—phubbing	0.167	0.029	0.111	0.224
Total		0.318	0.026	0.267	0.370

## Data Availability

The datasets used and analyzed during the current study are available from the corresponding author upon reasonable request.
